# Montreal Cognitive Assessment: Seeking a Single Cutoff Score May Not Be Optimal

**DOI:** 10.1155/2021/9984419

**Published:** 2021-09-25

**Authors:** Chongming Yang, Ling Wang, Hui Hu, Xinxiu Dong, Yuncui Wang, Fen Yang

**Affiliations:** ^1^Brigham Young University, Provo, UT, USA; ^2^Hubei University of Chinese Medicine, Wuhan, Hubei, China

## Abstract

**Background:**

Cutoff scores of the Montreal cognitive assessment (MoCA) for screening mild cognitive impairment in older adults differ across the world and within the Chinese culture. It is argued that to seek a cutoff score is essential to classify test participants. It was unknown how taking a classifying approach might reveal the cutoff score for identifying mildly cognitively impaired older adults.

**Methods:**

Participants, selected from 13 communities in Wuhan, China, were tested with the Chinese version of MoCA and rated with the Activities of Daily Living and the Clinical Dementia Rating scales. Mixture modeling was applied to the data with certain covariates and MoCA sum scores as the outcome of the latent class. Models with different numbers of classes were compared in terms of information criteria, likelihood ratio test, entropy, and interpretability.

**Results:**

A 3-class model (normal, mildly impaired, and severely impaired) was found to fit the data best. The normal class averaged a MoCA score of 24, while the severely impaired class averaged a score below 18. For those cases with MoCA scores above 18 and below 24, it is not certain if they are in the normal or the severely impaired classes.

**Conclusion:**

Latent variable classification modeling provides another option to identify MCI in older adults. Some categorically different cases of MCI cannot be captured with any single MoCA sum score. A range of 18–24 MoCA scores might serve as a better screening criterion of MCI. Older adults who scored within this gray zone should be monitored for potential interventions.

## 1. Introduction

The optimal cutoff score for screening mild cognitive impairment (MCI) in older adults has been widely explored in applying the Montreal Cognitive Assessment (MoCA), which is a tool designed exclusively for screening MCI in older adults [1]. Nevertheless, different from the original cutoff score of 24, various cutoffs have been identified, ranging from 18/19 to 26/27 across different cultures [2–6]. A recent meta-analysis of studies with strictly verifiable criteria of MCI suggested that the optimal cutoff was 23 based on balanced sensitivity (the probability of true positives) and specificity (the probability of true negatives) as well as samples of different language, cultural, and educational background. Unfortunately, only 86% cases could be correctly identified as either normal or MCI [7]. Recent studies in mainland China suggested that the cutoffs for MCI were 24 in a clinical sample [8] and ranged from 18 to 25 in normative samples [9–11]. These studies suggested that the cutoffs were contingent upon sampling (i.e., normative versus clinical), age, education, cultural background, and validating criteria [12]. Such inconsistency and contingency cast doubt on whether seeking a single cutoff score is an accomplishable goal and whether an alternative procedure might shed new light on any cutoffs.

A cutoff score has been typically determined according to the result of another gold standard validating criterion, which vary across studies. When applied to screening for MCI, a cutoff score indicates that participants above the cutoff score are classified as having normal cognition, and those below the cutoff score are considered cognitively impaired. In this sense, a cutoff score essentially creates a classification system for the test participants. Implementing a classification procedure might be more efficient than the typical approach and reveal the cutoff. In this methodological report, we briefly review the limitations of the typical approach of establishing a cutoff, introduce a mixture modeling for classification, and illustrate how classified participants mapped onto the MoCA sum scores.

Existing methods for setting cutoffs include experts' judgments [13], criterion or norm-referenced approaches [14], and statistical modeling [15]. In the criterion-referenced approach, the MoCA cutoffs are established in terms of other clinical standards and adjusted with the sensitivity and specificity from the receiver operating characteristic (ROC) analysis. Additionally, some studies have even adopted multiple standards to examine any cognitive impairment [16]. From the perspective of generalizability theory [17], it is advantageous to use multiple items/tasks, occasions, and raters to obtain a valid and generalizable measurement. However, a large variety of reference measures could lead to variations in cutoffs. For instance, sensitivity and specificity of the cutoff varied with the validating tools [12]. As such, there is no gold standard as to a cutoff score (i.e., validation criterion), as one scholar rather disappointingly stated: “There is no gold standard . . . not even a silver standard” [18].

Norm-referenced methods are subject to the characteristics of the norms. Large normative samples have yielded higher cutoffs than smaller normal or clinical samples [19, 20], but cutoffs also have to be lowered for lower educational attainment or older age [21]. Indeed, MCI could be complicated by underlying causes such as a lack of education, normal aging, or pathologic changes of the brain [22]. In the same logic, adjusting the cutoffs for other factors that affect cognitive functions would also be justifiable and likely to result in further cutoff variations. For instance, living alone increases the risk of developing dementia among the older adults with MCI by 50% [23, 24], while exercise improves global cognitive functions of older adults with MCI [25]. Thus, adjusting the cutoff for all important covariates could be necessary in the traditional approach, as doing so could lead to variations of the different cutoffs.

Model-based methods essentially use probabilistic models to link the probabilities of individuals' test responses to a hypothetical latent variable of cognitive ability. One of these models is latent class analysis (LCA), which assumes that individuals have categorically different abilities (referred to as latent classes) such as cognitively normal, mildly impaired, or severely impaired. In addition, covariates may be included in the model that affects the latent categorical variable [26]. LCA has been applied to identify profiles of cognitive impairment [27, 28] and has improved detection of early MCI and consequently the transition to dementia, compared to experts' judgment [29]. One limitation of LCA is that respondents are overrigidly presumed and restricted to having equal abilities within classes. In addition, class indicators (i.e., test items) with too many response categories make it difficult to interpret the class endorsement probabilities. However, this disadvantage can be overcome with a mixture model, which is introduced conceptually below.

Mixture modeling, also referred to as hybrid modeling, integrates item response theory (IRT) modeling with classification to score individuals on their latent abilities and to place them into different classes [30]. IRT essentially converts the test response patterns to individuals' continuous latent abilities based on a probabilistic distribution. Models may be selected to have different parameters such as item difficulty, discrimination, guessing, and so on [31]. A factor analysis model with categorical indicators of latent factors is essentially equivalent to IRT modeling with discrimination and difficulty parameters [32]. The advantage of factor analysis modeling of latent ability is that the sensitivity of each test item can be revealed in the factor loading [33].

Factor analysis modeling can be integrated with a latent profile analysis of the latent cognitive abilities and result in a mixture model. Mixture actually refers to hidden heterogenous distributions of individuals with similar abilities that can be identified with modeling. Essentially, the mean differences of the latent abilities are maximized across classes, while the variances are minimized within classes. Covariances of the latent ability variables may be fixed at zero or freely estimated [34]. This latent class variable can be predicted by other covariates using a multinomial logistic model. In addition, the latent class variable can also predict other outcome variables using another regression model. The optimal number of classes can be decided by comparing models of different numbers of classes in terms of information criteria, entropy, and loglikelihood test. The Bayesian Information Criteria (BIC) have performed well in identifying the number of classes for mixture modeling, where smaller BIC indicate a better fit model [35]. Compared to using scale sum scores of MoCA, which is weighted by the number of items in different cognitive domains, mixture modeling can include multiple measures and maximally use item information like difficulty (thresholds) and discrimination (factor loadings) and thus could be expected to improve classification and prediction [36–38].

It is also noteworthy to mention that setting a strict cutoff for cognitive test scores may not be an optimal goal, because such a dichotomization does not allow any probabilistic uncertainty. The underlying cognitive ability can be postulated to be a continuous random variable with a normal distribution, whose mean may be lower in older adults than in a normative population. As depicted in Figure 1, this normal distribution can be converted to a cumulative distribution, in which the horizontal axis indicates the underlying ability, and the vertical axis indicates the probability of one's ability in a population. For illustration, we have substituted and labeled the latent ability on the horizontal axis with the MoCA test scores based on the data of this study. As shown by the step function of the rectangle-marked line, a cutoff dichotomization implies a sharp qualitative difference in the latent ability on the two sides of the cutoff. Also, it is apparent that a single cutoff score does not capture the range of the MoCA scores around the cutoff. Thus, instead of a single cutoff, a range of MoCA scores might be plausible for identifying MCI.

There are some issues that arise when mixture modeling is applied to examine the cutoff of MoCA, such as how to incorporate potential validating measures. In order to attempt a better cutoff criterion for MoCA, we suggest using two of the many scales that have been referenced in studies assessing for MCI in Chinese cultural groups: the Activities of Daily Living (ADL) scale [39] and the Clinical Dementia Rating (CDR) scale [40]. The ADL assesses older adults' need for assistance [41], which in some cases may be due to MCI. Nygård suggested that Instrumental ADL should also be included in the diagnosis of MCI [42]. The CDR helps identify older adults with severely impaired cognitive functioning. We argue that the CDR and ADL are indispensable references for detecting MCI in older adults, because they differentiate normal functioning from cognitively impairment in older adults. We proposed a model as illustrated in Figure 2, in which scale items are linked to ADL, MoCA, or CDR through a factor analysis model. Covariates (rectangle at bottom-left) are linked to the class variable through multinomial logistic regression. The participants could be classified into various classes by the combination of their levels of three abilities measured with ADL, MoCA, and CDR through latent profile analysis model. MoCA sum scores were regressed on the class variable, however, without allowing it to affect the classifying process using a three-step approach [43]. Essentially, the three-step approach includes the following: (a) estimate the classes, (b) save the class membership, and (c) either regress the latent class variable on the covariates or use the latent class variable to further predict the outcomes. After the optimal numbers of classes are found in the estimation process, corresponding average levels of MoCA scores for all the classes are also ascertained. To the best of our knowledge, this is the first study to apply mixture modeling to identify the latent classes and then map the classes onto the MoCA sum scores to shed light on the cutoff. We hypothesized that three classes of the participants could be identified: cognitively severely impaired, mildly impaired, and normal in this sample. However, we could not clearly hypothesize how these three classes could be identified with the MoCA sum scores. For comparison, latent class analysis with covariates and a mixture model with only MoCA were also estimated to corroborate the advantage of mixture modeling.

## 2. Methods

### 2.1. Participants

The participants in this study (*n* = 697) were recruited from 13 urban communities in Wuhan, China, including Wuchang (zoned for culture and education), Hankou (zoned for commerce), and Hanyang (zoned for economic development). The sample consisted of five age groups: (1), 203 (29.1%) participants were 60–65 years old; (2) 151 (21.7%) were 65–69 years old; (3) 121 (17.4%) were 70–75 years old; (4) 135 (19.4%) were 76–80 years old; and (5) 87 (12.5%) were 80 years old or older. The distribution of participants' educational attainments was 14.6% illiterate; 22.4% elementary school; 33.7% middle school; 22.7% high school, vocational school, or technical school; and 6.6% associate's degree or above. Gender composition of the sample was 35.9% females (coded as 0) and 64.1% males (coded as 1). In addition, 14.8% of the sample were living alone (coded as 1, else = 0), and 46.5% had a disease history including one or more of the following: cerebrovascular disease, craniocerebral trauma, long-term diarrhea, thyroid syndrome, kidney diseases, carbon monoxide poisoning, and drug abuse. Some participants (13.8%) had family members with a history of vascular dementia, Alzheimer's disease, or mild cognitive impairment. A dichotomous variable of family history was defined for these cases (1 = true and 0 = false). Manual workers (coded as 1) and mental workers (coded as 0), respectively, accounted for 61.4% and 35.3% of participants' past careers (3.3% missing). This study purposely oversampled older adults in communities who might have experienced a decline in cognitive abilities, as described in the procedure below.

### 2.2. Procedure

Besides direct visits and invitations in the communities, researchers collaborated with community boards, medical station professionals, and enterprise human resources personnel on distributing paper notices, broadcasts, and social media messages about the study. Older adults who suspected that their memory was declining were encouraged and incentivized to participate in the research, with free gifts and medical services like massage, cupping, scraping, infrared heating, examinations, counseling, etc. Medical professionals and neurologists helped select participants who met the following criteria for the study: (1) ≥60 years old; (2) voluntary participation in the study; (3) no history of heart, liver, or kidney diseases; and (4) those who might have suspected problems with their memory or cognitive abilities. Data were collected through face-to-face interviews with demographics and the scales described below.

### 2.3. Measurement

Three scales (ADL, MoCA, and CDR) were used to interview the participants of the study. Original item scores of these were specified as ordinal indicators of latent factors (named as ADL, MoCA, and CDR), which were further specified as indicators of the latent classification variable “Class” (see Figure 2). Consequently, both continuous latent cognitive abilities and distinct classes were modeled based on probabilities of participants' responses, rather than the scale sum scores.

#### 2.3.1. Activities of Daily Living (ADL)

The ADL scale used in this study was mainly based on the Older American Resources and Services ADL scale [44]. Only one item of this scale (i.e., “get in and out of bed”) was replaced with an item (i.e., “laundry”) from the Lawton Instrumental ADL scale. ADL has a long developmental history and various versions with 3-point ratings [45] through 6-point ratings [46], but 4-point ratings capture more subtle differences than do 3-point ratings [47]. The Chinese version of this combined scale retained 4-point ratings: 1 = completely able to perform the activity, 2 = can perform the activity with some difficulty, 3 = can perform the activity but with some help, and 4 = completely unable to perform the activity. Higher scores indicate more help needed for the activities of daily living.

#### 2.3.2. Montreal Cognitive Assessment

Participants' cognitive functioning was assessed with the Chinese Beijing version of MoCA [7]. The Chinese Beijing version uses Chinese sequential characters and Arabic numbers, respectively, in place of the original English alphabets and requires participants to generate animal names instead of generating English words that start with a particular letter. High scores indicate more closeness to the normal cognitive function.

#### 2.3.3. Clinical Dementia Rating

The Chinese version of the CDR scale was adopted from the original CDR scale developed as a global rating device for a prospective study of mild senile dementia [48]. It was “found to distinguish unambiguously among older subjects with a wide range of cognitive functions, from healthy to severely impaired.” This study maintained the 5-level ratings (0 = healthy, 0.5 = questionable impairment, 1 = mild impairment, 2 = moderate impairment, 3 = severe impairment). Thus, higher scores indicate severe levels of dementia.

## 3. Analysis

The analysis was conducted in the following two steps. First, confirmatory factor analysis of the three scales was conducted to examine how well each item measured the latent abilities. The estimation method was weighted least squares estimation with Chi-square test and degrees of freedom adjusted for means and variances of the variables (WLSMV). Model fit is indicated by comparative fit index (CFI), Tucker-Lewis index (TLI), and root mean square errors of approximation (RMSEA). A model reflects data acceptably if CFI is close to 0.95, TLI is above 0.90, and RMSEA is below 0.08 and reflects data very well when CFI and TLI are close to 1.00, and RMSEA is close to 0.

Second, we estimated three mixture models of, respectively, 2, 3, and 4 classes. Each model included age, gender, education, exercise, living status, disease history, family history, and past career as covariates of the latent class variable and the MoCA sum scores as the outcome of the latent class variable (see Figure 2). The models were run in a 3-step approach, so that the MoCA sum score outcome was not allowed to affect the classifications, while yielding only its mean for each class. As the typical structural equation modeling fit indices no longer apply to mixture modeling, models with, respectively, 2, 3, and 4 classes were compared in terms of information criteria (i.e., Akaike [AIC], Bayesian [BIC], and sample-size adjusted Bayesian [ABIC]), likelihood ratio test (LRT), entropy, and the proportion of participants in the smallest class. Smaller information criteria indicate a better fit model. Likelihood Ratio Test compares *k* vs. *k* − 1 number of classes, with a significant *p* value indicating significant model difference. Entropy is a weighted average probability of participants in their primary classes. It ranges from 0 to 1, indicates less classification error when it is closer to 1 [49], and is preferred to be above 0.80 [50]. The proportion of participants in the smallest class is preferably above 5% [40]. However, the above information usually does not agree on the best number of class [51]. Therefore, in addition to these statistical indices, theoretical considerations, interpretability, and usefulness of the result are also important criteria when choosing the best model [52].

To compare and illustrate the advantage of mixture modeling, we also estimated a latent class analysis and a mixture model with only the MoCA scale. The results are presented in the following section in the above sequence. The analysis and modeling were primarily conducted with the advanced latent variable modeling software Mplus (8.4). Missing data were accounted for by the maximum likelihood estimation.

## 4. Results

### 4.1. Measurement Properties of the Scales

The confirmatory factor analysis indicated that the three scales measured three latent abilities well, with factor loadings ranging from acceptable (>0.40) to high. The standardized factor loadings are listed in Table 1. “Linking numbers and letters” and “orientation” of MoCA had the highest loadings, implying that older adults of this sample varied most in these two items compared to other items. Conceptually, these two items were the most sensitive in measuring the cognitive ability of the participants. Orientation in the CDR was also the most sensitive item as indicated by its highest factor loading. Factor loadings of the ADL items were all above 0.60, suggesting that those items measure the latent physical and cognitive abilities well. Some factor loadings were higher than 1.00, probably because those items had correlations with other items. No correlated residuals were estimated in the model, and the model fits the data acceptably (*χ*^2^_(461)_ = 1923.77, *p* < 0.01, CFI = 0.94, TLI = 0.93, RMSEA = 0.07). The reliabilities (*ω*) of the ADL, MoCA, and CDR were, respectively, 0.98, 0.89, and 0.82 [53].

### 4.2. Mixture Modeling of Three Scales with Covariates and Sum Scores as Outcomes

Information for three models, respectively, with 2 to 4 classes is listed in Table 2.

Based on the information criteria, entropy, likelihood ratio test, the smallest class proportion, and interpretability, we chose the first mixture model of ADL, MoCA, and CDR with 3 classes as the optimal result for the report. Other models of different classes had lower entropy, a nonsignificant LRT test, or overlarge proportions of participants that could not be interpreted as cognitively impaired in a normative community sample and thus are not further described or discussed in the study.

The profiles of the three classes of the chosen model are concisely expressed in the latent means of the three abilities measured with the three scales, as listed in Table 3. Class 3 served as the reference and had three means fixed at 0, because latent abilities in the population were treated as random variables with means of zero. As the scoring of MoCA is opposite to that of ADL and CDR, Class 3 with the highest level of MoCA and the lowest ADL and CDR was thus labeled as the “normal” group in Table 4. Class 1 with the highest levels of ADL and CDR but lowest level of MoCA was labeled as “severely impaired.” Class 2 included those who were intermediate in the three abilities and was labeled “mildly impaired.”

The covariate effects listed in Table 4 were obtained from the multinomial logistic regression portion of the model, with the latent class variable as the dependent and Class 3 as the reference. Compared to the normal reference (i.e., Class 3), males had 5.7 and 2.0 times higher odds of falling into classes 1 and 2 than females, respectively. For participants who aged 5 years older than others, their odds would increase 3.75 and 1.77 times to fall into classes 1 and 2, respectively. Participants who were one degree higher in education would have 11% and 27% lower odds to be in classes 1 and 2, respectively, as compared to the normal class. Manual workers also had 11% higher odds to be in the mildly impaired class, compared to the normal class. Disease history and family history, defined as in the participants section, did not affect the classification.

The predicted means of MoCA sum scores were 10.1 ± 0.9, 18.0 ± 0.4, and 24.4 ± 0.3 for the severely impaired, mildly impaired, and normal classes, respectively. The distributions of the MoCA scores are graphed for the three classes in Figure 3. Three vertical lines in the middle of the distributions indicate the MoCA means of the three classes. Figure 3 shows that participants who scored below 18.0 or above 24.0 in MoCA appeared to be, respectively, impaired or normal. In addition, participants of classes 2 and 3 overlap between the means of 18.0 and 24.4. The probability of being in the impaired class increases for those with lower scores, while the probability of being in the normal class increases for those with higher scores. However, participants with MoCA scores in this range have certain probabilities that can be classified as either mildly impaired (class 2) or normal (class 3).

## 5. Discussion

This study explored how distinct classes identified through mixture modeling would map onto the MoCA sum scores, so that a meaningful cutoff score might be revealed. We have postulated that using mixture modeling of multivariate cognitive test items is superior to the typical way that relies on certain validation standards and ROC analysis to determine the cutoff. The former identifies classes of participants using a probabilistic model, while the latter classifies participants according to the probabilities of meeting other criteria. This mixture modeling of ADL, MoCA, and CDR classified the participants into severely impaired, mildly impaired, and normal classes, while accounting for the effects of demographic covariates. Education and age affected the probability that a participant would belong to a certain Class. Mapping the three classes to the MoCA sum scores, we discovered that participants who scored either below 18 or above 24 were less prone to probabilistic errors to be cognitively impaired or normal, respectively. In contrast, it was difficult to differentiate whether participants were cognitively impaired or normal when they scored between 18 and 24 in MoCA. Thus, categorically different cases identified from the mixture modeling could not be clearly identified using any single MoCA cutoff score, implying that a range of scores had to be allowed for the purpose.

This wide range of MoCA scores (i.e., 18–24) for uncertain MCI from this study reflects the wide range of MoCA cutoffs found previous studies that used certain validating criteria and ROC analysis [2–12]. Studies that used latent class analysis also found cutoffs within a similar range, for instance, 19–25 [27] and 19–23 [28]. Therefore, whether using ROC analysis or latent variable classification, these studies suggested that a range of scores of MoCA scores for identifying MCI, depending on covariate adjustment, measures of cognitive ability, or sampling variations. For instance, our sample consisted of more participants who suspected memory or cognitive ability decline.

There may be two reasons for finding such a similar uncertainty in MoCA cutoffs. Statistically, classification through latent variable modeling is like using the step-function illustrated in Figure 1. Namely, more distinct classes would correspond to larger gray zones in the continuous MoCA. Further, it may be that the use of a cutoff score is a simplification of a complicated phenomenon and a suboptimal approach. Cognitive impairment is a latent status of brain function confounded with past education, age-related degeneration of physical functions, measurement errors due to test items and normal fluctuations of mental and physical functions, risk/protective factors of social life, nutrition, healthcare from a longitudinal perspective, etc. In this study, gender, education, age, and past career performing manual work were found to be important factors that affected the classification. This is consistent with previous studies that used education and age to adjust the sum score cutoffs [25]. Disease and family histories did not affect the classification, which might be explained as follows. Those above-mentioned diseases occurred in the remote past, they had not caused any brain damage, or the damage had recovered through the human self-healing ability. Participants with family members that had a history vascular dementia, Alzheimer's disease, or mild cognitive impaired were rare in this sample, and their hereditary linkages were not clearly probed in detail, annihilating any potential causality in this sample. We anticipated that our findings might change slightly if covariates and indicators of cognitive functions, other than those in this study, were incorporated into the model.

Questions remain as to whether we should designate the cutoff as 18, 24, somewhere in between, or abandon the pursuit of a single cutoff altogether. It proved to be counterproductive to seek a single MoCA cutoff to determine a latent status affected by so many factors. Further efforts in the typical approach are likely to find a cutoff within a certain range. We suggest that clinical professionals adopt a range of 18–24 of the MoCA scores, instead of single cutoff, as a screening threshold of MCI for determining appropriate diagnosis and treatments.

This study has the following limitations. First, biochemical and neural function measures were not collected and included in the model. Second, there was no follow-up measurement to determine any cognitive deterioration or progression to dementia that could further validate the classification. Third, as our sample is a nonnormative community sample, it is unknown how findings of this study may generalize to a normative community sample. Future studies may take similar approach to validate our findings.

Methodologically, the analysis that involves classification of individuals has been referred to as the person-centered approach, which has advantages of identifying individuals with similar characteristics and has become a useful tool for studying cognitive impairment. As latent classification techniques are increasingly used to identify typological individuals [42, 54, 55], future research may adopt mixture modeling with a biopsychosocial perspective and incorporate blood test, biomarkers, or neuroimaging, and neuropsychological measures to improve classification accuracy. Researchers may also consider longitudinal designs and optimal temporal intervals for repeated measurement, so that changes can be observed.

In conclusion, classification based on latent variable modeling is another way to identify cognitively impaired older adults. To continue to use the sum scores of MoCA, it is recommended that a score range of 18–24 may be adopted for professionals to monitor the cognitive functions of older adults and provide appropriate interventions.

## Figures and Tables

**Figure 1:** Three hypothetical functions of MoCA.

**Figure 2:** Illustration of the mixture model with covariates and MoCA sum scores as outcomes of latent classes.

**Figure 3:** Distributions of MoCA sum scores of three classes.

**Table 1:** Standardized factor loadings of three scales.

Activities of daily living		Montreal cognitive assessment		Clinical dementia rating	
Item content	Factor loading	Item content	Factor loading	Item content	Factor loading
Taking transportation	0.75	Linking numbers and letters	0.89	Memory	0.55
Walking	0.62	Copy cubes	0.74	Orientation	0.94
Preparing meals	0.89	Drawing clock	0.66	Judgment and problem solving	0.52
Doing housework	0.90	Naming	0.54	Community affairs	0.64
Taking own medications	0.83	Repeat list of digits	0.47	Home and hobbies	0.48
Eating	1.09	Repeat digits and knocking	0.55	Personal care	0.75
Dressing and undressing	0.88	Subtraction of 7	0.65		
Taking care of appearance	0.98	Repeat sentence	0.48		
Doing laundry	0.77	Fluency (words)	0.64		
Bathing/showering	1.10	Abstraction	0.65		
Shopping for groceries	0.80	Delayed recall	0.53		
Getting to bathroom on time	0.82	Orientation	0.85		
Using telephone	0.94				
Handling finances	0.78				

**Table 2:** Information for models of 2–4 classes.

Model	Classes	AIC	BIC	ABIC^a^	Entropy	LRT *p*	Smallest class %
(1) Mixture modeling of ADL, MoCA, and CDR	2	19770	20319	19932	0.87	<0.00	36.6
	**3**	**19365**	**19964**	**19541**	**0.83**	**<0.01**	**13.1**
	4	19249	19897	19400	0.79	0.68	2.5
(2) Mixture modeling of only MoCA	2	12642	12867	12708	0.83	<0.00	37.2
	3	12362	12628	12441	0.78	<0.01	18.1
	4	12286	12592	12376	0.80	<0.01	3.6
(3) Latent class analysis of only MoCA	2	12635	12941	12725	0.84	<0.00	37.7
	3	12390	12867	12531	0.82	0.76	14.8
	4	12348	12996	12539	0.78	0.79	12.0

Note. LRT = likelihood ratio test of *k* vs. *k* − 1 number of classes.

**Table 3:** Latent means of abilities and proportions of three classes.

Latent factor	Class 1 (13.1%, *n* = 87) severely impaired	Class 2 (41.3%, *n* = 275) mildly impaired	Class 3 (45.6%, *n* = 304) normal
MoCA	−4.76^*∗∗*^ [−6.41, −3.12]	−2.46^*∗∗*^ [−3.23, −1.68]	0
ADL	2.92^*∗∗*^ [1.91, 3.94]	0.41 [−0.95, 1.77]	0
CDR	2.50^*∗∗*^ [1.74, 3.26]	1.07^*∗∗*^ [0.65, 1.50]	0

^*∗∗*^, *p* < 0.01 (estimate is significantly different from zero).

**Table 4:** Covariate effects on latent class in odds ratios and 95% confidence interval [LL, UL].

Covariates	Severely impaired		Mildly impaired	
	Coefficients	Odds ratios	Coefficients	Odds ratios
Gender	1.74^*∗∗*^ [0.73, 2.75]	5.70 [2.08, 15.59]	0.70^*∗∗*^ [0.11, 1.28]	2.00 [1.12, 3.60]
Age	1.32^*∗∗*^ [0.90, 1.74]	3.75 [2.47, 5.70]	0.57^*∗∗*^ [0.32, 0.82]	1.77 [1.38, 2.26]
Living alone	−0.20 [−1.24, 0.83]	0.82 [0.29, 2.30]	−0.35 [−1.25, 0.56]	0.71 [0.29, 1.75]
Manual worker	−0.47 [−1.44, 0.49]	0.62 [0.24, 1.63]	−0.89^*∗*^ [−1.57, −0.21]	0.41 [0.21, 0.81]
Education	−2.20^*∗∗*^ [−2.89, −1.51]	0.11 [0.06, 0.22]	−1.32^*∗∗*^ [−1.66, −0.97]	0.27 [0.19, 0.38]
Having dis. his.	−0.30 [−1.08, 0.47]	0.74 [0.34, 1.65]	−0.37 [−0.95, 0.21]	0.69 [0.39, 1.23]
Having fam. his.	−0.88 [−2.15, 0.39]	0.41 [0.12, 1.48]	−0.47 [−1.23, 0.28]	0.62 [0.29, 1.33]

LL = lower limit; UL = upper limit; ^*∗*^*p* < 0.05;  ^*∗∗*^*p* < 0.01; living status = living alone or not; dis. his = disease history; Fam. his = family history; Manual = manual worker (1) vs. mental worker (0).

## Data Availability

All data included in this study are available upon request to the corresponding author.
